# Effects of neuromuscular electrical stimulation on exercise capacity and quality of life in COPD patients: a systematic review and meta-analysis

**DOI:** 10.1042/BSR20191912

**Published:** 2020-05-27

**Authors:** Xu Wu, Xianglin Hu, Weiping Hu, Guiling Xiang, Shanqun Li

**Affiliations:** Department of Pulmonary Medicine, Zhongshan Hospital, Fudan University, Shanghai 200032, China

**Keywords:** Chronic obstructive pulmonary disease, Exercise capacity, Life quality, Neuromuscular electrical stimulation, Pulmonary rehabilitation

## Abstract

Neuromuscular electrical stimulation (NMES) has been shown to produce benefits in the muscle function of chronic obstructive pulmonary disease (COPD) patients. The definite effectiveness of NMES, applied in isolation or concurrently with conventional pulmonary rehabilitation (PR) or exercise training, remains unclear. This review was to determine the effects of NMES on exercise capacity, functional performance, symptoms, and health-related quality of life (HRQoL) in COPD patients. Electronic databases (PubMed, Embase, Web of Science, the Cochrane Library) were searched for relevant randomized controlled trials (RCTs). Two investigators independently screened the eligible studies up to February 2020 that used NMES as the intervention group. The outcome measures were 6-min walking distance (6MWD), peak rate of oxygen uptake (VO_2_ peak), St George’s Respiratory Questionnaire (SGRQ), and symptoms of dyspnoea and fatigue. Data were extracted using a predefined table and papers were appraised using Downs and Black tool. We analyzed 13 RCTs with 447 COPD patients. In the analysis of 6MWD, pooled estimates showed a significant increase in the NMES group, compared with the control group (mean difference (MD) = 27.05, 95% confidence interval (CI): 8.46–45.63, *P*<0.001). There were also improvements in symptoms of dyspnea or leg fatigue, and reduction in London Chest Activity of Daily Living (LCADL) scores. No statistically significant difference was observed in VO_2_ peak, peak power, and SGRQ. NMES could improve exercise capacity and reduce perceived sensation of dyspnea during exercise in patients with COPD, but not to be recommended as an effective alternative training modality in the rehabilitation of stable COPD patients.

## Background

Chronic obstructive pulmonary disease (COPD) is a systemic disease that is characterized by incompletely reversible airflow obstruction [1]. It is widely known that numerous COPD patients suffer from locomotor disorder and dysfunction [2]. As the most common extrapulmonary manifestation of COPD, progressive skeletal muscle impairment leads to decreased strength, endurance, exercise tolerance and in turn, a poor prognosis [3]. Moreover, muscle wasting and resting dyspnea, as well as greater fatigue during exercise are observed. It has been well documented that pulmonary rehabilitation (PR) is safe and beneficial to increase exercise capacity and peak oxygen consumption [4]. As the most important component of the PR programs, physical exercise training is performed to improve the functional capacity in COPD patients. Numerous studies have confirmed that severe COPD patients cannot undergo physical training due to advanced heart failure or respiratory failure, which progressively impedes performance of physical exercise.

Passive training of targeted muscle groups with the use of neuromuscular electrical stimulation (NMES) is a valuable intervention strategy to depolarize the motor neurons and induce involuntary muscle contractions [5]. The clinical benefits of NMES has been widely reported in the improved muscle function of COPD patients. Particularly, there is a 20–30% gain in quadriceps strength as compared with control subjects, usual care or sham stimulation, which indicates that NMES is a potential adjunctive technique, especially for patients who abandon physical exercise because of the discomfort related to dyspnea.

In recent decades, most consistent findings of NMES training have supported the beneficial effects on COPD patients, lately, Bonnevie et al. have revealed that unsupervised home-based NMES as an add-on to PR does not further improve benefits in subjects with severe to very severe COPD [6]. What is worse, it might be a burden for some subjects. Pan et al. pooled randomized controlled trials (RCTs) into the analysis and found NMES might not be effective in improving quadriceps muscle strength, exercise capacity, and muscle fiber characteristics [7]. Most RCT studies have small sample sizes and different outcome measures, and thus convey inconclusive results. Therefore, we searched the newest literature, performed a meta-analysis, and critically assessed the effects of NMES, applied in isolation or concurrently with conventional PR or exercise training, on the exercise capacity, functional performance, symptoms, and health-related quality of life (HRQoL) in patients with COPD.

## Methods

We used the Preferred Reporting Items for Systematic Reviews and Meta-Analyses (PRISMA) 2009 checklist to report the review [8].

### Literature search strategy and selection criteria

A computerized search was performed through PubMed, Web of Science, Embase, Cochrane Central Register of Controlled Trials (upto February 2020) to detect RCTs. We used the following combined text and Medical Subject Headings (MeSH) search terms ‘chronic obstructive pulmonary disease’, ‘neuromuscular electrical stimulation’. Studies were filtered for human subjects and published trials written in English. We excluded randomized crossover trials. The inclusive selection criteria were: (i) age ≥ 18 with confirmed diagnosis of severe or very severe stable COPD, at least during recruitment, participants in the present study were clinically stable; (ii) the objective of the research was to compare the NMES with usual care (any aspect of usual medical care, with or without sham training, or conventional exercise training), or PR (exercise training); (iii) useful outcomes of RCTs.

### Outcomes

The primary outcome was exercise capacity which mainly referred to 6-min walk distance (6MWD), peak rate of oxygen uptake (VO_2_ peak), and peak power. The secondary outcomes were HRQoL (using validated St George’s Respiratory Questionnaire (SGRQ)); symptoms of dyspnea and fatigue (using any validated questionnaire or scale). The London Chest Activity of Daily Living (LCADL) scale evaluates dyspnea-related functional impairment, it is frequently used to analyze dyspnea limitation during exercises and activities of daily living (ADL) accomplishment in COPD patients.

### Data extraction

Two investigators (X.W. and S.Y.H.) independently extracted and assessed eligibility, data, and trial quality information from the selected papers for inclusion in the meta-analysis. We extracted the following study characteristics, including author’s name, year of publication, study design, participants and control group information, sample size, duration of intervention, intervention protocol and outcomes.

### Quality assessment

The methodological quality assessment was evaluated. The risk of bias was assessed using Downs and Black tool. Two authors (X.W. and X.L.H.) reviewed all the studies and evaluated each study in accordance with the 27-point tool assessing studies in five key sections: (i) study quality (10 points), (ii) external validity (3 points), (iii) study bias (7 points), (iv) confounding and selection bias (6 points), and (v) power of the study (1 point).

### Statistical analysis

Meta-analyses were done with RevMan 5.3 software (Cochrane Collaboration, London, U.K.). For continuous outcomes, differences were expressed as weighted mean difference (MD) or standardized MDs with 95% confidence intervals (CI). *I^2^* statistic was used to measure statistical heterogeneity across studies in each analysis. Studies with *I^2^* < 25% have low heterogeneity, *I^2^* of 25–75% indicates medium heterogeneity, and *I^2^* > 75% implies high heterogeneity. We explored possible causes of substantial heterogeneity (*I^2^* of 50% or greater) through sensitivity analyses. We conducted sensitivity analyses by excluding studies that described the use of different methodologies. A *P*-value less than 0.05 for all outcome measures were considered to be statistically significant.

## Results

### Literature retrieved and study characteristics

The search strategy yielded 197 potential studies, of which 43 were duplicates that were removed as part of the electronic search process. Of the 154 remaining potential studies, 89 records were excluded based on title or abstract and 42 studies were excluded after reading the full paper. Of the 23 RCT studies, 5 studies were excluded for the participants who were recruited during hospitalization for an exacerbation. Although the recruited participants were once ventilated via a tracheostomy for chronic respiratory failure in the study by Zanotti et al., at the time of recruitment, participants were clinically stable [9]. However, we excluded this study for the lack of useful outcomes to extract in the review. Finally, 13 studies involving a total of 447 patients (NMES vs control: 233 vs 214) were included in the meta-analyses. A flow chart for the screened studies and the exclusion reasons is shown in Figure 1.

**Figure 1:** Flow of study selection in different phases of the meta-analysis

The main characteristics of the 13 RCTs are presented in Tables 1 and 2. Of the 13 studies that met the inclusion criteria, 7 studies explored the effect of NMES versus usual care [10–16,17]. This comparison allowed us to determine the effects of NMES in isolation from other exercise rehabilitation strategies. On the other hand, six studies compared NMES plus conventional exercise training versus exercise training alone, with or without sham training NMES [6,14,18,19,34,35]. This comparison allowed us to determine the effects of using NMES as an adjunct to conventional PR.

**Table 1:** Basic characteristics of the researches included

Investigator	Study design	Study group	Control group	Group size	Participants
Daniel, 2020	Prospective, RCT	NMES + PR (treadmill, stationary bicycle, quadriceps resistance training, and breathing exercises)	PR without any stimulation	NMES + PR (*n*=19); PR (*n*=19)	Clinically stable COPD, males, 40–75 years, eligibility to participate in exercise training, no acute exacerbations within 3 months
Mekki, 2018	RCT	NMES + PR (comprised motion, stretching, low-intensity aerobic exercises, ergocycle, and interset break)	PR without NMES	NMES + PR (*n*=25); Control (*n*=20)	COPD and post-bronchodilator results on spirometry of forced expiratory volume in 1 s/forced vital capacity < 0.7
Valenza, 2018	RCT	Standard medical treatment + standard rehabilitation program with superimposed NMES	Standard medical treatment based on long-acting bronchodilators without any physical therapy	NMES group (*n*=18) Control group (*n*=18)	Stable severe COPD age ranging from 40 to 80 years
Bonnevie, 2018	Single-blind, multicenter randomized trial	PR+NMES group underwent bilateral NMES of the quadriceps muscle at home	Comprehensive PR program (outpatient or home-based) including respiratory physiotherapy, and strength and endurance training on a cycloergometer	PR+NMES (*n*=27) PR (*n*=24)	Severe COPD with forced expiratory volume in 1 s < 60% predicted with a total lung capacity > 80% predicted; baseline modified Medical Research Council dyspnea scale > 1; aged ≥ 18 years
Maddocks, 2016	Double-blind randomized, randomized trial	NMES group received electrical stimulation of the quadriceps of both lower limbs	Placebo NMES (I: 0–20 mA), insufficient to elicit a tetanic muscular contraction	NMES group (*n*=25) Control group (*n*=27)	18 years or older, with a spirometrically defined diagnosis of COPD consistent with GOLD criteria (forced expiratory volume in 1 s:forced vital capacity [FEV1:FVC] < 70%), severe respiratory impairment (FEV1% predicted ≤ 50), and incapacitating breathlessness
Kucio, 2016	RCT	NMES + PR (comprised breathing exercises, treadmill walking and resistance exercise)	PR for 3 weeks without stimulation	NMES + PR (*n*=15); PR (*n*=15)	Hospitalized participants: 11 men, mean FEV1 = 1.66 (SD: 0.69) L, mean age = 68 (SD: 6) yr
Tasdemir, 2015	Double-blind randomized, randomized trial	NMES + cPR (program for 2 days per week over 10 weeks)	cPR: mainly exercise training. Sham NMES using a similar protocol, and the intensity was sufficient to cause a visible twitch muscular contraction	NMES + cPR (*n*=13); cPR (*n*=14)	Medically stable COPD (median FEV1% predicted = 29 (range: 16–71) %, mean age = 62 (SD: 8) yr)
Vieira, 2014	Double-blind randomized, randomized trial	NMES + respiratory physical therapy (i.e., airway clearance)	Respiratory physical therapy + sham NMES (same instruction and electrode position, but no stimulation)	NMES (*n*=11); control (*n*=9)	Medically stable COPD (mean FEV1% predicted = 36 (SD: 10) %, mean age = 56 (SD: 11) yr)
Sille, 2014	Prospective, single-blind, RCT	HF-NMES	Strength training (bilateral leg extension and bilateral leg press exercises)	HF-NMES (*n*=41); control (*n*=40)	Not provided
Vivodtzev, 2012	Double-blind RCT	NMES group (bilateral electrical stimulation of the quadriceps (35 min) followed by bilateral stimulation of the calf muscles)	Sham training: the same fashion (5 Hz of frequency in the continuous mode with a 100-μs pulse duration)	NMES (*n*=12); Control (*n*=8)	Medically stable COPD (mean FEV1% predicted = 34 (SEM: 3) %, mean age = 70 (SEM: 1) yr)
Vivodtzev, 2006	Single-blind RCT	NMES (bilateral electrical stimulation of both quadriceps) + rehabilitation 4 days per week for 4 weeks, which comprised active limb exercises	Rehabilitation without any stimulation	NMES + UR (*n*=9); UR (*n*=8)	Medically stable COPD (mean FEV1 = 27 (SD: 3) % predicted, mean age = 59 (SD: 15) yr)
Neder, 2002	Double-blind RCT	NMES (electrical stimulation of both quadriceps)	Usual care, NMES after a control period of 6 week	NMES (*n*=9); Control (*n*=6)	Medically stable COPD (mean FEV1% predicted = 38 (SD: 10) %, mean age = 67 (SD: 8) yr)
Bourjeily-Habr, 2002	Double-blind double-blind controlled trial	NMES (electrical stimulation of the hamstrings, quadriceps and calf muscles of both lower limbs)	Sham stimulation same electrode, without any active electrical stimulation	NMES (*n*=9); Control (*n*=9)	Medically stable COPD (mean FEV1% predicted = 36 (SEM: 4) %, mean age = 58 (SEM: 2) yr)

**Table 2:** Characteristics of interventions for the researches included

Investigator	Intervention duration	Intervention parameters	Outcomes
Daniel, 2020	4 weeks, 5 sessions/week, 60 min/session	Frequency: 20–35 Hz; pulse duration: NR, intensity: 15–90 mA; duty cycle: NR	SGRQ, mMRC, spirometry, PImax, PEmax, 6MWT, bio-electrical impedance
Mekki, 2018	24 weeks, three times per week, 45 min underwent the same endurance training and 20 min of NMES	Frequency: 50 Hz; pulse duration: 400 μs; intensity: 15–60 mA; duty cycle: 5 s on/15 s off during the first 3 months and 10 s on/30 s thereafter	A stabilometric platform, time up and go, Berg balance scale tests, 6MWT, the maximal voluntary contraction
Valenza 2018	8-week: 1 h twice a week (2 h/week). Ten minutes of warm-up; 30 min of NMES superimposed on to voluntary muscular contraction; 5 min of relaxation/cool down	Frequency: 50 Hz; pulse duration: 400 ms; the contraction time was 8 s with 20 s of relaxation	SGRQ; 6MWT; 5STS; controlling heart rate (HR), respiratory rate (RR), dyspnea; leg fatigue; FIM; LCADL scale
Bonnevie, 2018	8 weeks: 5 times per week; 30 min of stimulation	Pulse duration: 400 ms; 10 min of warm-up at 6 Hz, the intensity was individually adjusted to just under the pain threshold. The frequencies used were 35 Hz for the contractions and 4 Hz for the active rest phases, with a duty cycle of 0.5 and 1.5 s for 25 min. Three-minute recovery period at 3 Hz	6MWT; VO_2_ peak; maximal workload during CPET; Dyspnea; BMI; airflow obstruction; exercise capacity index, and HRQoL, including SGRQ subscores
Maddocks, 2016	6 week × 7 sessions/week; 30 min/per session	Frequency: 50 Hz; pulse duration: 350 μs; intensity: max tolerable; duty cycle: 2 s on/15 s off to 10 s on/15 s off	6MWT; quadriceps muscle strength (MVC); fat-free mass via bioimpedance physical activity; SGRQ
Kucio, 2016	Not provided	NMES of the quadriceps and gastrocnemius using symmetric rectangular impulses with pulse width of 0.30 ms at a frequency of 35 Hz for 2 s on and 4 s off for 36 min	6MWT; airflow obstruction; arterial oxygen and carbon dioxide concentrations
Tasdemir, 2015	10 week × 2 sessions/week; 20 min/per session	Frequency: 50 Hz; pulse duration: 300 μs; intensity: max individual tolerance (29.43–35.81 mA); duty cycle: 10 s on/20 s off	SWT; dyspnoea; quadriceps muscle strength; exercise endurance; MRC; SGRQ LCADL; feelings of anxiety and depression
Vieira, 2014	8 week × 5 sessions/week; 60 min/per session	Frequency: 50 Hz; pulse duration: 300–400 μs; intensity: max tolerable (15–20 to 100 mA); duty cycle: 2 s on/18 s off to 10 s on/30 s off	Thigh circumference; 6MWT; VO_2_ peak and endurance time; dyspnea; muscle activity; SGRQ; fat-free mass; respiratory muscle strength
Sillen, 2014	8 week × 5 sessions/week; 18 min/per session	Frequency: 75 Hz; pulse duration: 400 μs intensity: max tolerable; duty cycle: not provided	Quadriceps muscle strength (isokinetic quadriceps muscle strength); constant work-rate cycling endurance test; 6MWT; exercise endurance; dyspnea; SGRQ
Vivodtzev, 2012	6 week × 5 sessions/week; 35 min of stimulation of the quadriceps followed by 25 min of stimulation of the calf/per session	Frequency: 50 Hz; Pulse duration: 400 μs; Intensity: NR; Duty cycle: 2 s on/16 s off	Quadriceps strength and endurance; incremental and endurance shuttle walk test with cardiorespiratory monitoring; muscle signaling pathways, enzyme activity, fiber type and size, and capillarization via biopsy
Vivodtzev, 2006	4 week × 4 sessions/week; 30 min/per session	Frequency: 35 Hz; pulse duration: 400 μs; intensity: max tolerable (21–46 mA); duty cycle: 47%	Airflow obstruction via spirometry; BMI; Quality of life and dyspnoea; Respiratory failure questionnaire; Quadriceps muscle strength; Quadriceps muscle composition
Neder, 2002	6 week × 5 sessions/week; 15 min/per session for the first week, after 30 min/per session	Frequency: 50 Hz; pulse duration: 300–400 μs; intensity: 10–20 to 100 mA; duty cycle: 2 s on/18 s off to 10 s on/30 s off	Quadriceps strength (peak torque), exercise endurance; cardiopulmonary exercise test; HRQoL; lung volumes and airflow obstruction
Bourjeily-Habr, 2002	6 week × 3 sessions/week; 20 min/per session	Frequency: 50 Hz; pulse duration: NA; intensity: 56.7–95 mA; duty cycle: 0.2 s on/1.3 s off	SWT; quadriceps strength (isokinetic peak torque); cardiopulmonary exercise test

Abbreviations: cPR, comprehensive PR; FEV1, forced expiratory volume in 1 s; FIM, functional independence measure; MRC, Medical Research Council scale; MVC, maximum voluntary contraction; SWT, shuttle-walk test; UR, usual rehabilitation; 5STS, five-times-sit-to-stand test; 6MWT, 6-min walk test.

### Primary outcomes

Overall, patients in the NMES intervention group showed a significant improvement of 27.1 m compared with the control group in a pooled analysis of nine studies (*n*=367), as shown in Figure 2. Meta-analysis of these studies demonstrated a high statistical heterogeneity (*I^2^* = 86%). Thus, a subgroup analysis was undertaken according to the study group. Of these, four studies that compared NMES with usual care reported on the assessment of 6MWD. The pooled MDs from these studies were 20.5 m (95% CI: −0.57 to 41.56, *P*=0.06). Besides, five studies demonstrated a between-group difference in favor of NMES plus conventional exercise training on 6MWD (MD: 36.64 m; 95% CI: 22.15–51.13, *P*<0.00001), did reach the statistical significance. These data suggested that the gains in exercise capacity may have been greater following an NMES training when compared with the control group.

**Figure 2:** Meta-analysis of the effect of NMES on 6MWD in COPD patients

Three studies on 83 participants examined the effects of experimental group versus control on peak power. However, there was a trend in favor of control group (MD: −1.43; 95% CI: −2.6 to −0.25, *P*=0.02; Figure 3). The results were not consistent in these RCTs when evaluating the mean value of peak power. Rather than performing a subgroup analysis for the NMES effect on peak power based on the study group, we undertook a sensitivity analysis. After excluding the study by Bonnevie et al. [6], the pooled MD was 5.77 (95% CI: −6.00 to 17.53; participants = 33), indicating favoring the NMES group. It was suggested that the control group demonstrated an improvement in VO_2_ peak compared with NMES group (MD: −1.09, 95% CI: −2.10 to −0.08; *P*=0.03), as shown in Figure 4. Although both studies included in this meta-analysis showed the different direction of effect, this analysis had no statistical heterogeneity (*I^2^* = 0%). In the study conducted by Bonnevie et al., the PR alone led to a mean improvement of VO_2_ peak after rehabilitation (15.8 ml/kg/min; *P*=0.04) [6]. When we excluded this study, the MD from the remaining four studies was 61.57 (95% CI: −30.63 to 153.78; participants = 73), but the difference was not significant.

**Figure 3:** Meta-analysis of the effect of NMES on peak power in COPD patients

**Figure 4:** Meta-analysis of the effect of NMES on VO_2_peak in COPD patients

As modified Medical Research Council Scale assesses functional limitation resulting in dyspnea rather than the severity of dyspnoea itself [20], grade from the study by Bonnevie et al. [6] was not included in the assessment of leg fatigue. Five studies used the Borg 0–10 scale to evaluate changes in leg fatigue at the end of an exercise test. The symptoms of leg fatigue were significantly relieved (MD: −1.14, 95% CI: −1.42 to −0.86, *P*<0.00001; Figure 5) after intervention. These trials showed heterogeneity when they were pooled in a meta-analysis (*I^2^* = 79%). However, there were sufficient studies to undertake planned subgroup analyses for the effect on leg fatigue based on the study group. Pooled analysis showed that NMES group was associated with a statistically significant improvement in reported dyspnoea at the end of an exercise test using the Borg 0–10 scale (MD: −0.45, 95% CI: −0.66 to −0.24; *P*<0.00001; Figure 6). In the five studies that compared NMES with usual care alone, the pooled effect size showed that the NMES group had a lower dyspnea score than the usual care group (MD: −1.17, 95% CI: −2.14 to −0.21; *P*<0.00001). However, heterogeneity was also high among the five trials (*I^2^* = 89%). In five studies that compared NMES plus conventional PR training with PR alone, the NMES plus PR training group showed a significantly decreased dyspnoea scores (MD: −0.37, 95% CI: −0.59 to −0.16; *P*<0.001) compared with the exercise group.

**Figure 5:** Meta-analysis of the effect of NMES on leg fatigue in COPD patients

**Figure 6:** Meta-analysis of the effect of NMES on dyspnoea in COPD patients

### Secondary outcomes

Regarding the assessment of HRQoL, six studies used the SGRQ. Pooled analysis of these studies showed no difference between groups using a fixed-effects model (MD: −0.39, 95% CI: −0.93 to 0.16; *P*=0.17); however, there was inconsistency between individual studies with high heterogeneity (*I^2^* = 78%). Furthermore, for this sensitivity analysis, if the study by Sillen et al. [10] was excluded, heterogeneity was markedly abated (*I^2^* = 57%) as shown in Figure 7. These data suggested that the score of the SGRQ was higher following an NMES training when compared with the control group.

**Figure 7:** Meta-analysis of the effect of NMES on SGRQ in COPD patients

In the LCADL, patients showed an improvement of −5.35 (95% CI: −8.86 to −1.83; *P*=0.003; Figure 8) in the NMES group compared with the control group in a pooled analysis of two studies (*n*=63). Of note, this analysis had high statistical heterogeneity (*I^2^* = 92%).

**Figure 8:** Meta-analysis of the effect of NMES on LCADL in COPD patients

### Risk-of-bias and quality assessment

Table 3 shows the assessment of the included studies using Downs and Black tool.

**Table 3:** Down and Black quality assessment

	Daniel (2020)	Mekki (2018)	Valenza (2018)	Bonnevie (2018)	Maddocks (2016)	Kucio (2016)	Tasdemir (2015)	Vieira (2014)	Sillen (2014)	Vivodtzev (2012)	Vivodtzev (2006)	Neder (2002)	Bourjeily- Habr (2002)
Hypotheses/aims/objectives clearly described	√	√	√	√	√	√	√	√	√	√	√	√	√
Main outcome measures clearly described	√	√	√	√	√	√	√	√	√	√	√	√	√
Characteristics of patients/subjects clearly described	×	√	√	√	√	√	√	√	×	√	√	√	√
Interventions of interest clearly described	√	√	√	√	√	√	√	√	√	√	√	√	√
Distribution of principal confounders in each group clearly described	×	√	√	√	√	×	√	√	√	√	×	√	×
Main findings clearly described	√	√	√	√	√	√	√	√	√	√	√	√	√
Estimates of random variability in the data provided	×	√	√	√	√	×	√	√	√	×	×	×	×
Important adverse events reported	N/A	N/A	N/A	N/A	N/A	N/A	N/A	N/A	N/A	N/A	N/A	N/A	N/A
Characteristics of patients lost to follow-up described	N/A	N/A	N/A	N/A	N/A	N/A	N/A	N/A	N/A	N/A	N/A	N/A	N/A
Actual probability values reported	√	√	√	√	√	√	√	√	√	√	√	√	√
Participants approached representative of entire population	√	√	√	√	√	√	√	√	√	√	√	√	√
Participants recruited representative of entire population	√	√	√	√	√	√	√	√	√	√	√	√	√
Staff, places, and facilities were patients treated representative of majority of population	√	√	√	√	√	√	√	√	√	√	√	√	√
Blinding of study subjects	N/A	N/A	N/A	N/A	N/A	N/A	N/A	N/A	N/A	N/A	N/A	N/A	N/A
Blinding of assessors	×	√	√	N/S	×	N/S	N/S	N/S	×	N/S	N/S	N/S	N/S
Data based on data-dredging clearly stated	N/A	N/A	N/A	N/A	N/A	N/A	N/A	N/A	N/A	N/A	N/A	N/A	N/A
Time period between the intervention and outcome the same for cases and controls	N/A	N/A	N/A	N/A	N/A	N/A	N/A	N/A	N/A	N/A	N/A	N/A	N/A
Appropriate statistical tests used	√	√	√	√	√	√	√	√	√	√	√	√	√
Compliance to intervention reliable	N/A	N/A	N/A	N/A	N/A	N/A	N/A	N/A	N/A	N/A	N/A	N/A	N/A
Main outcome measure reliable and valid	√	√	√	√	√	√	√	√	√	√	√	√	√
Intervention groups or case–controls recruited from same population	√	√	√	√	√	√	√	√	√	√	√	√	√
Intervention groups or case–controls recruited at the same time	√	√	√	√	√	√	√	√	√	√	√	√	√
Study subjects randomized to the interventions	×	√	√	N/S	×	×	×	×	×	×	N/S	×	×
Was concealed randomization to allocation undertaken	N/A	N/A	N/A	N/A	N/A	N/A	N/A	N/A	N/A	N/A	N/A	N/A	N/A
Adequate adjustment made in the analysis of confounders	√	√	√	√	√	√	√	√	√	√	√	√	√
Patient losses accounted for	N/A	N/A	N/A	N/A	N/A	N/A	N/A	N/A	N/A	N/A	N/A	N/A	N/A
Sufficiently powered cohort size	√	√	√	√	√	√	√	√	√	√	×	×	×

Abbreviations: N/A, not applicable; N/S, not stated.

Studies included in this meta-analysis had clear hypothesis, outcome measures and aims (*n*=13, 100%). The outcome measures were reliable and clearly reported (*n*=13, 100%) with sufficiently powered cohort size (*n*=10, 76.9%). Particular limitations were that assessors were not blinded (*n*=1, 7.7%) and estimates of random variability was present in only half of studies (*n*=7, 53.8%).

## Discussion

The primary findings of the present study were that NMES promoted a significant increase in exercise tolerance measured with the 6MWT, and such changes were accompanied by improvements in symptoms of dyspnoea and fatigue, increase in SGRQ scores and reduction in LCADL scores. It needs to be highlighted that, the beneficial effect of 6MWT was lessened when this intervention was combined with conventional exercise training or applied alone. Nevertheless, no statistically increase in HRQoL was noted among participants allocated with NMES. Our results also showed that NMES had no benefit for the VO_2_ peak and peak power. The results of our study are in accordance with the study by Pan et al. that there was insufficient evidence to support the positive effects exerted by NMES in COPD patients.

Physical exercise capacity is the core content of the rehabilitation in clinically stable severe COPD patients. 6MWD has been used as a simple and valid evaluation indicator for exercise tolerance of COPD patients [21]. A previous review reported a significant increase in walking distance was larger than that seen in the current review (MD: 37.27 m) [22]. In our pooled analysis of all the studies, NMES significantly increased the 6MWD, but not all statistically significant differences are clinically relevant when interpreting clinical measures. The mean 6MWD changes were 27.05 m among the clinically important difference (minimum clinically important difference (MCID)) ranging from 25 to 33 m [23].

As compared with conventional exercise training, the major advantage of NMES in patients with COPD is the virtual absence of ventilatory stress during passive exercise. It does not provoke dyspnea for severely disabled patients with COPD, and also can be used at home. NMES has the potential to break the vicious circle of negative emotions, unpleasant respiratory sensations, furthermore, the smaller muscle mass involved improves exercise capacity and quality of life. To date, the additional benefit of adding NMES to a comprehensive PR program remains debated.

In the study by Dal Corso et al., no significant increase in distance walked in the 6MWT in the NMES group patients was noted [24]. Our estimated effects of NMES in addition to a comprehensive PR program have reached statistical significance, which were been assessed in five randomized studies. Kaymaz et al. suggested that NMES could be used as an effective treatment strategy in PR programs for peripheral muscle training in patients with severe COPD [25]. But they showed no further benefits when NMES was added to a comprehensive PR program regarding the walking distance, endurance time, the MRC, and HRQoL [25].

Regarding other measures of exercise capacity, VO_2_ peak appeared to be not improved in all pooled studies except for one study, although the treatment response was not heterogeneous. This result was not consistent with earlier review that demonstrated a significant increase in VO_2_ peak [26]. In addition, dyspnea is a critical factor in restricting exercise performance. Most patients with COPD present peripheral muscle fatigue associated with intensive dynamic hyperinflation [27]. Earlier work suggested that NMES reduced dyspnoea, but did not separate the studies that applied NMES in isolation from those that applied NMES plus conventional exercise training.

A negative effect of NMES on the aspect of HRQoL was observed. Our results are in line with previous meta-review [22], in which pooled estimates showed NMES may reduce HRQoL measured by the SGRQ with high heterogeneity. This heterogeneity was probably due to the fact that the SGRQ was influenced by many other factors [28]. Nevertheless, it contrasts with a retrospective and observational study that demonstrated NMES significantly improved the overall HRQoL in patients with COPD, regardless of the severity of airflow obstruction [29].

The improved exercise performance could be attributed to the stimulation intensity, subsequent gains in quadriceps strength and reduced ventilatory demand during walking [5]. Meanwhile, it depends on patients’ progression in the PR program and the reported levels of fatigue and dyspnea. Some reviews combined data across only three to five studies, whose results were inconsistent, thus resulting in low precision for our estimate of the effect. As to the outcomes related to functional performance, symptoms and HRQoL, our results showed high levels of heterogeneity. The disparity can be explained by several reasons. Our findings in the meta-analysis appear to have been influenced by the inclusion of a study. Apparently, the NMES protocols included in this review were diverse. Specifically, a difference in parameters of stimulation could influence the potential response [30]. The observed changes were correlated with a progressive increase in the used electrical stimulation [31]. But there were insufficient studies to determine the most effective protocol. Also, the interpretation of our results should take into account the severity of initial impairment. As suggested by their different response to exercise stimulation [32], patients with severe to very severe COPD might achieve their maximal possible improvement from either NMES alone or PR alone. In contradiction to the aforementioned studies, Wedzicha et al. reported that patients with less severe respiratory disease might experience further benefits with additional NMES [33].

The fundamental limitation of the meta-analysis was that the quality of the evidence was very low, and largely limited by poor methodology, at least in part, leading to the risk of bias. Additionally, in contrast with the previous meta-analysis, current review did not measure the muscular physiological changes. Based on current available data, NMES should not be regarded as a replacement for PR completely, for the combination does not result in further improvement. It is worth noting that, for the participants who are unable or unwilling to attend PR programs, consideration could be given to using NMES.

## Conclusions

In conclusion, our meta-analysis involved large numbers of patients with 13 RCTs, and extended previous finding by suggesting that, NMES was effective in improving exercise capacity, but the true effect on this outcome measure could be trivial. As expected, functional capacity of the patients could be enhanced, which was indicated by an improvement in dyspnea sensation during ADL. Future studies should add the data describing the intrinsic muscle function or peripheral muscle force, and following up the adverse signs or events, in which NMES is applied alone or in isolation from rehabilitation strategies. High quality of the evidence that assess the underlying physiological mechanisms and explore the optimal NMES training regimen are also warranted.

## Abbreviations

6MWD: 6-min walk distance
ADL: activities of daily living
CI: confidence interval
COPD: chronic obstructive pulmonary disease
HRQoL: health-related quality of life
LCADL: London Chest Activity of Daily Living
MD: mean difference
NMES: neuromuscular electrical stimulation
PR: pulmonary rehabilitation
RCT: randomized controlled trial
SGRQ: St George’s Respiratory Questionnaire
VO_2_ peak: peak rate of oxygen uptake
